RETRACTED

# The melanocortin signaling cAMP axis accelerates repair and reduces mutagenesis of platinum-induced DNA damage

**DOI:** 10.1038/s41598-017-12056-5

**Published:** 2017-09-15

**Authors:** Stuart G. Jarrett, Katharine M. Carter, Brent J. Shelton, John A. D’Orazio

**Affiliations:** 1 The Markey Cancer Center, University of Kentucky College of Medicine, Lexington, Kentucky 40536 USA; 2 Department of Toxiciology and Cancer Biology, University of Kentucky College of Medicine, Lexington, Kentucky 40536 USA; 3 Department of Cancer Biostatistics, University of Kentucky College of Medicine, Lexington, Kentucky 40536 USA; 4 Department of Pediatrics, University of Kentucky College of Medicine, Lexington, Kentucky 40536 USA

## Abstract

Using primary melanocytes and HEK293 cells, we found that cAMP signaling accelerates repair of bi- and mono-functional platinum-induced DNA damage. Elevating cAMP signaling either by the agonistic MC1R ligand melanocyte stimulating hormone (MSH) or by pharmacologic cAMP induction by forskolin enhanced clearance of intrastrand cisplatin-adducts in melanocytes or MC1R-transfected HEK293 cells. MC1R antagonists human beta-defensin 3 and agouti signaling protein blocked MSH- but not forskolin-mediated enhancement of platinum-induced DNA damage. cAMP-enhanced repair of cisplatin-induced DNA damage was dependent on PKA-mediated phosphorylation of ATR on S435 which promoted ATR’s interaction with the key NER factor xeroderma pigmentosum A (XPA) and facilitated recruitment of an XPA-ATR-pS435 complex to sites of cisplatin DNA damage. Moreover, we developed an oligonucleotide retrieval immunoprecipitation (ORiP) assay using a novel platinated-DNA substrate to establish kinetics of ATR-pS435 and XPA’s associations with cisplatin-damaged DNA. Expression of a non-phosphorylatable ATR-S435A construct or deletion of A kinase-anchoring protein 12 (AKAP12) impeded platinum adduct clearance and prevented cAMP-mediated enhancement of ATR and XPA’s associations with cisplatin-damaged DNA, indicating that ATR phosphorylation at S435 is necessary for cAMP-enhanced repair of platinum-induced damage and protection against cisplatin-induced mutagenesis. These data implicate cAMP signaling as a critical regulator of genomic stability against platinum-induced mutagenesis.

## Introduction

There are more than fifteen million cancer survivors in the United States^1^. Platinum-based agents are important components of a variety of multimodal oncologic treatment regimens because they interfere with replication and DNA homeostasis by altering the structure of nucleotides and DNA. Though platinum compounds are useful in treating a variety of cancers, they promote genomic instability and mutagenesis by chemically modifying nucleic acid bases. Consequently, development of secondary malignancies is a well-characterized long-term risk of platinum exposure. Survivors of childhood cancers are at particularly high risk for secondary malignancies because many patients survive their primary cancers and there is ample latency time to develop secondary malignancies because of their young age when exposed to chemotherapy^2,3^. In fact, melanoma is among the most common secondary tumors among childhood cancer survivors, occurring 14 times more frequently than in an age-matched cohort not exposed to chemotherapy^4^. One retrospective meta-analysis concluded that melanoma accounts for 5.3% of all secondary cancers among survivors of pediatric malignancies, with survivors of Hodgkin disease, hereditary retinoblastoma and soft tissue sarcomas especially at risk (standardized incidence ratios of 6.7, 27.6 and 6.7, respectively)^5^. Since platinum-based therapeutics are commonly used to treat childhood malignancies, we posit that a critical determinant of secondary melanoma risk may be the capacity of melanocytes to repair platinum-induced DNA injury and that sub-optimal repair would favor mutagenesis and genomic instability. Hence, a greater understanding of the biochemical mechanisms that promote cisplatin-repair/resistance is important for predicting the likelihood for the development of secondary malignancies and for developing useful melanoma-preventive approaches in high-risk patients.

RETRACTED

The melanocortin 1 receptor (MC1R) is a highly polymorphic G_s_ protein-coupled cell surface receptor on melanocytes^6^ that functions as a global regulator of melanocyte physiology and damage responses^7,8^. When stimulated by its agonistic ligand MSH, MC1R promotes the formation of the second messenger cAMP through activation of adenylyl cyclase^9^. MC1R signaling is impacted by a variety of ligands which regulate MC1R-cAMP responses. Agouti signaling protein (ASIP) functions as an inverse agonist for MC1R decreasing MC1R basal signaling^10^ while human β-defensin 3 (HBD3) is a neutral antagonist that blunts effects of other MC1R ligands^11,12^. In humans, *MC1R* is highly polymorphic with more than 70 variants, many of which impair MC1R-cAMP signaling responses^13^. At least five “red hair color” (RHC) single nucleotide polymorphisms (MC1R-D84E, -R142H, -R151C, -R160W, and -D294H) are associated with red hair, freckling, fair skin, UV sensitivity and increased lifetime melanoma risk^6^.

We and others have reported that MC1R/cAMP signaling regulates melanocyte genomic stability by enhancing and accelerating nucleotide excision repair (NER)-mediated clearance of helix-distorting, replication-blocking DNA adducts generated by UV^14–19^. Like UV, cisplatin damages DNA in ways that interfere with replication, transcription and genomic stability. The major effect cisplatin has on DNA is to generate intrastrand adducts by forming covalent bonds with the N^7^ position of adjacent purine bases to form 1,2- or 1,3-intrastrand crosslinks. Intrastrand platinum-induced DNA adducts distort the double helix and are recognized and removed by NER^20^. The xeroderma pigmentosum complementation group proteins (XPs), which include XPA through XPG, play a critical role in coordinating and promoting NER^21–23^. XP group A (XPA) deficiency exhibits among the highest UV sensitivity among XP cells^24,25^. Functionally, XPA is involved in many steps of NER including DNA damage verification, stabilization of repair intermediates and positioning NER factors appropriately at sites of action^26,27^. Similarly, ATR is critical to UV DNA damage signaling^28^ and is linked with NER^29–34^. Furthermore, ATR provides an anti-mutagenic role in a subset of melanomas^35^. We recently described a molecular pathway linking MC1R signaling with XPA through a protein kinase A (PKA)-mediated phosphorylation event on ATR at S435, which accelerates the repair of UV-induced DNA damage^19^.

RETRACTED

The role of MC1R signaling in the repair of cisplatin-induced DNA damage is unknown but has clear implications for predicting secondary melanoma risk after platinum chemotherapy. Because of the significance of MC1R-directed NER in the repair of UV damage in melanocytes^19,36,37^, we reasoned that MC1R/cAMP signaling may regulate cellular recovery from platinum-induced DNA injury. Herein, we report that cAMP enhances melanocyte responses to platinum-induced DNA damage through PKA-mediated ATR phosphorylation on S435 and subsequent accelerated recruitment of XPA to nuclear cisplatin damage. Moreover, cAMP stimulation diminished levels of cisplatin-mediated mutagenesis suggesting that the MC1R-cAMP signaling axis is a master regulator of genomic stability in melanocytes. A greater understanding of how genomic stability is regulated in platinum-exposed melanocytes may inform novel approaches to enhance repair in *MC1R*-defective, melanoma-susceptible individuals or for purposely impairing repair to enhance platinum-chemotherapeutic effects.

## Results

### MC1R/cAMP signaling enhances the repair of cisplatin-induced DNA damage

To determine whether cAMP signaling affected repair of DNA damage caused by platinum-based chemotherapeutics, we measured DNA repair kinetics in HEK293 cells pre-treated with either vehicle or forskolin, an adenylyl cyclase activator that induces a strong cAMP signal independently of MC1R status. To directly compare the cAMP-influence on repair of platinum-induced DNA damage, a panel of three bi-functional (cisplatin, oxaliplatin and carboplatin) and one monofunctional (phenanthriplatin) compounds were administered to HEK293 cells, and DNA repair measured by XL-PCR detecting PCR-based amplification of a 5 kb fragment of the hypoxanthine guanine phosphoribosyl transferase (*HPRT)* gene. In this assay, presence of DNA damage interferes with polymerase amplification of the target sequence. As cells repair the damage, there is proportionally more amplification of the sequence^38^. Although repair kinetics differed between platinum agents, forskolin pre-treatment significantly increased repair kinetics for all platinum agents (Fig. 1), supporting the hypothesis that cAMP signaling accelerates clearance of platinum DNA adducts. Intriguingly, repair kinetics were faster among three bi-functional platinum agents (cisplatin, carboplatin and oxaliplatin) when compared to clearance of the mono-functional agent (phenanthriplatin), suggesting that the higher degree of distortion of the double helix caused by intrastrand purine adducts is more efficiently recognized and repaired by NER as compared to monoadducts^38^. We compared cAMP-mediated augmentation of repair between UV injury in PHMs from our previous studies^19,39^ to cisplatin repair in the current study. We observed that cAMP increased repair kinetics for either UV photoproducts or intrastrand cisplatin-adducts (pt-GpGs), but the extent of repair enhancement varied depending on the DNA lesion (6.3-fold cAMP boost for pt-GpG, 2.1-fold cAMP boost for 6-4-PP, and 1.7-fold cAMP boost for CPDs). We then focused our attention on the mechanisms of cAMP-enhanced repair of cisplatin-mediated DNA injury since cisplatin is a mainstay of a variety of anticancer chemotherapeuitic regimens^40^ and signaling mechanisms controlling the repair of its genomic toxicity are poorly understood. Thus, we determined whether MC1R signaling influenced repair efficiency of cisplatin-mediated DNA damage. We measured cisplatin repair kinetics in primary human melanocytes (PHMs) as well as HEK293 cells transfected with either wild type (*MC1R* ^*WT*^) or loss-of-function MC1R (*MC1R* ^*R151C*^). MSH treatment of cells expressing functional MC1R (PHM and HEK293-MC1R-WT) resulted in significantly increased repair efficiency compared to vehicle (Table 1 and Fig. S1). HEK293 cells transfected with signaling defective MC1R (*MC1R* ^*R151C*^), in contrast, demonstrated a markedly blunted DNA repair response to MSH (Table 1 and Fig. S1). Forskolin enhanced clearance of cisplatin adducts in all cell lines irrespective of MC1R status (Table 1 and Fig. S1). To determine the biological consequence of MC1R in the removal of cisplatin-damaged DNA, we tested the ability of its natural antagonistic ligands to regulate NER. Co-treatment of PHMs with MSH and either HBD3, a neutral MC1R antagonist^11,12^, or ASIP, an inverse MC1R antagonist^10^, blocked MSH-mediated augmentation of cisplatin repair (Table 1 and Fig. S1). Neither HBD3 nor ASIP interfered with forskolin-mediated enhanced repair (Table 1 and Fig. S1), consistent with MC1R-independent generation of cAMP by direct activation of adenylyl cyclase by the drug. Importantly, the presence of MC1R did not appear to impact cellular sensitivity to cisplatin in HEK293 cells (Fig. S2). Together, these data strongly support an integral role for MC1R/cAMP to accelerate clearance of platinum DNA adducts and support the hypothesis that pharmacologic induction of cAMP signaling enhances NER.

RETRACTED

**Figure 1:** cAMP signaling enhances the repair of platinum-induced DNA damage. HEK293 cells were pre-treated with either forskolin (10 µM), or vehicle (1% EtOH) for 30 minutes before (**A**) cisplatin, (**B**) carboplatin, (**C**) oxaliplatin, (**D**) phenanthriplatin treatment (100 µM each) for 1 hr. DNA repair was determined at 3 and 9 hr post-damage by measuring amplification by XL-PCR of a 5 kb fragment of the *HPRT* gene. Efficiency of PCR amplification between damage and control samples was used to calculate repair at each time point. Repair levels in forskolin treated cells significantly different from vehicle at indicated time points were determined by 2-way ANOVA (*p ≤ 0.05). Data are expressed as mean ± SEM from three independent experiments.

**Table 1:** cAMP enhances the repair of cisplatin-induced DNA damage.

Cell line	Treatment	Repair half time (minutes)
PHM	*Vehicle*	*421* ± 31^*a*^
	*MSH*	*114* ± 16^*b*^
	*HBD3* + *MSH*	*423* ± 27^*a*^
	*ASIP* + *MSH*	*434* ± 17^*a*^
	*Vehicle*	*387* ± 31^*a*^
	*forskolin*	*61* ± 23^*b*^
	*HBD3* + *forskolin*	*76* ± 18^*b*^
	*ASIP* + *forskolin*	*69* ± 13^*b*^
HEK293-MC1R-WT	*Vehicle*	*452* ± 32^*a*^
	*MSH*	*123* ± 16^*b*^
	*HBD3* + *MSH*	*482* ± 21^*a*^
	*ASIP* + *MSH*	*472* ± 18^*a*^
	*Vehicle*	*462* ± 0.3^*a*^
	*Forskolin*	*65* ± 17^*b*^
	*HBD3* + *forskolin*	*67* ± 21^*b*^
	*ASIP* + *forskolin*	*69* ± 26^*b*^
HEK293-MC1R-R151C	*Vehicle*	*462* ± 12^*a*^
	*MSH*	*462* ± 15^*a*^
	*HBD3* + *MSH*	*412* ± 24^*a*^
	*ASIP* + *MSH*	*427* ± 33^*a*^
	*Vehicle*	*372* ± 31^*a*^
	*forskolin*	*68* ± 16^*b*^
	*HBD3* + *forskolin*	*62* ± 21^*b*^
	*ASIP* + *forskolin*	*71* ± 18^*b*^

Primary human melanocytes (PHM), HEK293-MC1R-WT or HEK293-MC1R-R151C cells were pre-treated with either MSH (100 nM), MSH (100 nM) + ASIP (100 nM) or HBD3 (100 nM) or forskolin (10 µM), forskolin (10 µM) + ASIP (100 nM) or forskolin (10 µM) + HBD3 (100 nM), 30 minutes before cisplatin (100 µM) or mock treatment for 1 hr. Following which, the repair of intra-strand DNA damage was monitored using an anti-pt-GpG antibody. Repair efficiencies are expressed as time taken in hours to repair 50% of initial damage and expressed as mean ± SEM. Values not sharing a common letter were significantly different for each treatment (per cell type) as determined by one-way ANOVA; p ≤ 0.05. Data are expressed as mean ± SEM from three independent experiments.

RETRACTED

### MC1R-cAMP signaling enhances the kinetics of ATR-pS435 generation following cisplatin-induced DNA damage

As cAMP-mediated enhancement of NER active against UV is dependent on phosphorylation of ATR on the S435 residue^19^, we posited that cAMP-mediated acceleration of platinum damage repair was similarly dependent on PKA-mediated generation of ATR-pS435. We previously established that ATR-pS435 accumulation was dependent not only on cAMP induction but also on UV damage, suggesting cooperation between MC1R signaling and cellular damage responses. Therefore, we explored enzyme kinetics of S435 phosphorylation in platinum-damaged cells activated by cAMP signaling. To determine this, we utilized a high-throughput screening method using a biotinylated peptide containing ATR-S435 and a phosphospecific anti-ATR-pS435 antibody^39^. Even though this assay does not take into account full-length ATR and structural contributions to the S435 phosphorylation events, it permits interrogation of rapid phosphorylation kinetics at the repair-relevant residue (e.g. S435). We compared the ability of PHMs and HEK cells transfected with *MC1R* ^*WT*^ or *MC1R* ^*R151C*^ to generate ATR-pS435 in the presence or absence of cisplatin. All lines demonstrated decreased *K*_m_ values as well as elevated V_max_ levels of ATR-S435 phosphorylation when exposed to cisplatin and induced by cAMP. ATR-pS435 generation occurred in response to MC1R signaling as demonstrated by robust induction of MC1R-intact cells treated with either MSH or forskolin (Table 2 and Fig. S3). cAMP-induced enhancement of ATR-pS435 was further validated by Western blotting, as demonstrated by elevated levels of this phosphorylation event (Fig. S3). MC1R-dependence of ATR-pS435 was demonstrated by observing the lack of induction by MSH in cisplatin-exposed MC1R-defective cells or in MSH-treated and cisplatin-exposed *MC1R* ^*WT*^ cells co-incubated with either ASIP or HBD3 (Table 2 and Fig. S3). Neither ASIP nor HBD3 impacted forskolin-mediated generation of ATR-pS435 in cisplatin-treated cells (Table 2 and Fig. S3), suggesting that ASIP and HBD3 antagonize MSH-MC1R interactions rather than inhibit downstream cAMP responses such as PKA-mediated ATR phosphorylation. Together, these data suggest that cisplatin-induced melanocyte damage responses cooperate with MC1R/cAMP signaling to promote ATR-pS435 accumulation and resultant enhanced NER activity.

RETRACTED

**Table 2:** cAMP enhances ATR-pS435 generation following cisplatin damage.

Cell line	Cisplatin treated	Treatment	V_max_	K_m_
PHM	−	*Vehicle*	*n*.*d*.	*n*.*d*.
	+	*Vehicle*	*10* ± 4	*31* ± 3
	+	*MSH*	*24* ± 3	19 ± 6
	+	*HBD3* + *MSH*	*11* ± 2	*33* ± 4
	+	*ASIP* + *MSH*	*n*.*d*	*n*.*d*.
	−	*Vehicle*	*n*.*d*.	*n*.*d*.
	+	*Vehicle*	*13* ± 4	*31* ± 4
	+	*Forskolin*	*29* ± 4	3 ± 2
	+	*ASIP* + *Forskolin*	*31* ± 5	4 ± 2
	+	*HBD3* + *Forskolin*	*28* ± 5	5 ± 3
HEK293 (MC1R-WT)	−	*Vehicle*	*n*.*d*.	*n*.*d*.
	+	*Vehicle*	*9* ± 4	*28* ± 4
	+	*MSH*	*23* ± 4	19 ± 4
	+	*HBD3* + *MSH*	*13* ± 2	*33* ± 3
	+	*ASIP* + *MSH*	*n*.*d*	*n*.*d*.
	−	*Vehicle*	*n*.*d*.	*n*.*d*.
	+	*Vehicle*	*11* ± 2	*24* ± 6
	+	*Forskolin*	*32* ± 5	5 ± 2
	+	*HBD3* + *Forskolin*	*34* ± 5	6 ± 3
	+	*ASIP* + *Forskolin*	*26* ± 6	7 ± 3
HEK293 (MC1R-R151C)	−	*Vehicle*	*n*.*d*.	*n*.*d*.
	+	*Vehicle*	*11* ± 3	*23* ± 7
	+	*MSH*	*12* ± 5	*21* ± 5
	+	*HBD3* + *MSH*	*9* ± 4	*24* ± 6
	+	*ASIP* + *MSH*	*n*.*d*.	*n*.*d*.
	−	*Vehicle*	*n*.*d*.	*n*.*d*.
	+	*Vehicle*	*16* ± 2	*26* ± 4
	+	*Forskolin*	*32* ± 5	5 ± 2
	+	*HBD3* + *Forskolin*	*28* ± 3	6 ± 3
	+	*ASIP* + *Forskolin*	*26* ± 6	5 ± 2

Cell lysates were extracted from either primary human melanocytes (PHM), HEK293-MC1R-WT or HEK293-R151C, following pre-treatment with either forskolin (10 μM), MSH (100 nM) or vehicle for 30 minutes followed by 1 hr cisplatin exposure (100 μM). ATR-pS435 was measured using the peptide CPKRRRLSSSLNPS (10 μM) as a substrate for 3 minutes (phosphorylation of the substrate was linear within this period). Kinetic parameters of the phosphorylation reaction were calculated by nonlinear regression analysis for the oligopeptide substrate using anti-ATR-pS435 antibody coupled with colorimetric detection. “n.d.” = none detected (below the limits of detection).

### MC1R-cAMP signaling enhances the interactions of XPA, ATR, and AKAP12 with cisplatin-damaged chromatin

To obtain insight into the mechanism by which cAMP impacts repair of cisplatin-mediated DNA damage, we tested the impact of cAMP stimulation to influence binding of XPA, ATR and A kinase anchoring protein 12 (AKAP12), three key proteins involved in cAMP-enhanced repair of UV damage^19,39,41^, to cisplatin-damaged DNA. Treatment of PHMs and *MC1R* ^*WT*^-transfected HEK293 cells with MSH significantly increased levels of chromatin-bound ATR, XPA and AKAP12 (Fig. 2). None of these proteins interacted with chromatin isolated from cells not exposed to cisplatin. Inclusion of either ASIP or HBD3 abrogated MSH-mediated (but not forskolin-induced) benefit, confirming the importance of MC1R in MSH-directed enhancement of ATR, XPA and AKAP12 binding to cisplatin-damaged DNA and the ability of pharmacologic cAMP induction to circumvent MC1R antagonism. To further confirm the specificity and importance of MC1R, studies were performed in MC1R-wild type or -mutant (*MC1R* ^*R151C*^-transfected) HEK293 cells. MSH pre-treatment failed to influence binding of XPA, ATR, or AKAP12 to cisplatin-damaged DNA in mutant but not wild type cells. Forskolin enhanced levels of XPA, ATR and AKAP12 in all cell lines irrespective of the MC1R status or presence of MC1R-antagonists. Furthermore, the enhanced cAMP-protein levels appear to be specific to ATR, XPA and AKAP12, as levels of XPC and CSB, two other NER factors, were not modulated by forskolin pre-treatment (Fig. S4).

RETRACTED

**Figure 2:** MC1R-cAMP signaling enhances chromatin-bound protein levels of ATR, XPA and AKAP12 following cisplatin treatment. (**A**) Wild-type primary human melanocytes (PHM). (**B**) *MC1R* ^*WT*^-expressing HEK293 cells or (**C**) *MC1R* ^*R151C*^-expressing HEK293 cells were pre-treated with either forskolin (10 µM), MSH (100 nM), MSH (100 nM) + ASIP (100 nM) or MSH (100 nM) + HBD3 (100 nM) 30 minutes before cisplatin (100 µM) or mock treatment for 1 hr. Chromatin extracts were isolated and probed for either anti-XPA, anti-ATR, anti-AKAP12 or anti-H2A by Western blotting. ATR and XPA bands were cropped from the same blot. AKAP12 bands were cropped from a separate blot.

### MC1R-cAMP signaling enhances XPA-, ATR-, and AKAP12-DNA interactions following cisplatin-induced DNA damage

To explore the potential kinetic parameters of MC1R/cAMP-enhanced binding of XPA, ATR and AKAP12 to cisplatin-damaged DNA, we adapted the “oligonucleotide retrieval assay-immunoprecipitation” (ORiP) assay^39^ to measure protein-cisplatin-damaged DNA interactions. This assay takes advantage of a biotinylated and cisplatin-damaged oligonucleotide to identify proteins associated with cisplatin damage. Briefly, nuclear lysates are isolated and incubated with a cisplatin-damaged oligonucleotide that is retrieved by streptavidin; bound proteins are identified using antibodies and colorimetric detection. In this way, we measured levels of oligonucleotide-bound XPA, ATR, ATR-pS435 and AKAP12 in nuclear lysates of either HEK293 cells transfected with wild-type MC1R or the R151C mutant variant and pre-treated as indicated (Fig. 3). In *MC1R* ^*WT*^-expressing cells, pre-treatment with MSH or forskolin promoted binding of XPA, ATR-pS435 and AKAP12 to the damaged oligonucleotide substrate roughly 3–4 fold above vehicle (*p* ≤ 0.05) up to 30 min post-damage (Fig. 3A,B and C). Incubation with either ASIP or HBD3 reduced MSH-induced association of all factors with the damaged oligonucleotide substrate up to 30 min post-damage (i.e. not cAMP stimulated) (Fig. 3A,B and C) and each was significantly reduced compared to MSH alone (*p* ≤ 0.05). We observed essentially no interaction with either XPA, ATR-p435S or AKAP12 with undamaged oligo substrate, irrespective of MSH or forskolin treatment. Considering a longer time course post-damage, we observed that extent of XPA-binding to the damaged-oligonucleotide returned to basal levels at 4 h in unstimulated cells. In contrast, forskolin pre-treatment resulted in an XPA-oligonucleotide interaction that remained elevated above baseline through 4 h (Fig. S5). Furthermore, Western blots confirmed that forskolin enhanced binding of XPA to cisplatin-damaged chromatin over the same time course as that observed by ORiP (Fig. S5).

RETRACTED

**Figure 3:** MC1R-cAMP signaling enhances interactions between XPA, ATR-pS435 and AKAP12 to a cisplatin-damaged substrate by ORiP. *MC1R* ^*WT*^- or *MC1R* ^*R151C*^-expressing HEK293 cells were pre-treated with either forskolin (10 µM), MSH (100 nM), MSH (100 nM) + ASIP (100 nM) or MSH (100 nM) + HBD3 (100 nM) 30 minutes before cisplatin treatment (100 µM) for 1 hr. Isolated nuclear extracts were incubated with a cisplatin-damaged DNA fragment (which acts as a substrate for NER) for a period of 30 minutes at 30 °C, as described in the Experimental Procedures. The interaction with the DNA substrate with (**A**) XPA, (**B**) ATR-pS435, (**C**) AKAP12 were determined using antibodies and quantified as described in Experimental Procedures for ORiP. Data are expressed as mean ± SEM from three independent experiments.

To determine the importance of ATR-pS435 in the recruitment of these factors to cisplatin-induced DNA damage, a knock-down and rescue approach was employed. Endogenous ATR was suppressed and HEK293 cells were transfected with siRNA-resistant S435 wild type or S435A ATR constructs (Fig. 4). Rescue with wild type S435 ATR promoted cAMP-enhanced binding of XPA, ATR, ATR-pS435 or AKAP12 to cisplatin-damaged DNA. In stark contrast, expression of the non-phosphorylatable ATR-S435A abolished any benefit of MSH-MC1R-cAMP signaling on protein-DNA interactions (Fig. 4). None of these proteins interacted with the DNA substrate from cells not exposed to cisplatin (Fig. S6). To directly determine the importance of ATR-pS435 in the repair of cisplatin-induced DNA damage, we again utilized a knock-down and rescue approach. Native ATR was suppressed in HEK293 cells and cells were transfected with siRNA-resistant S435 wild type or S435A ATR constructs. We found that forskolin accelerated repair of cisplatin damage in S435-WT but had no effect in S435A ATR-transfected cells (Fig. S7). Since our previous work established that PKA-mediated ATR phosphorylation (on S435) is scaffolded by AKAP12^41^, we tested the contribution of AKAP12 to cAMP enhancement of cisplatin repair in HEK293 cells with endogenous AKAP12 knocked down by siRNA. Transfection of an siRNA-resistant wild type AKAP12 permitted cAMP enhancement of cisplatin repair whereas transfection of a PKA binding-defective AKAP12 mutant^41^ abrogated any forskolin-induced benefit on the repair of cisplatin-induced DNA damage (Fig. S8). Together, these data suggest a role for ATR-pS435 in the recognition and repair of cisplatin DNA damage.

RETRACTED

**Figure 4:** cAMP-induced phosphorylation of ATR at S435 is critical to enhanced interactions of XPA, ATR and AKAP12 to a cisplatin-damaged substrate. HEK293 cells were treated with siRNA-directed to ATR, and then transfected with either (**A**,**B**) siRNA-resistant ATR-WT or (**C**,**D**), siRNA-resistant ATR-S435A Cells were pre-treated with forskolin (10 μM; 30 min) or vehicle and exposed to cisplatin (100 µM) for 1 hr. Lysates were incubated with a cisplatin-damaged ORiP substrate for protein-DNA binding analysis as described in Experimental Procedures. Data are expressed as mean ± SEM from three independent experiments.

### MC1R/cAMP signaling promotes association of XPA with ATR-pS435 on cisplatin-damaged DNA

As XPA is indispensable for NER^42^ and since phosphorylation of ATR at S435 enhances NER by recruiting XPA to UV-induced DNA damage^19^, we wished to determine how cAMP and physiologic MC1R ligands impacted ATR-pS435-XPA recruitment to cisplatin-damaged DNA. We found that cAMP signaling enhanced levels of ATR-pS435 in cisplatin-damaged chromatin in *MC1R* ^*WT*^-expressing cells treated with MSH compared to vehicle alone (Fig. S9). Incubation with either ASIP or HBD3 antagonized MSH’s enhancement of ATR-pS435 (Fig. S9). Additionally, proximity ligation in *MC1R* ^*WT*^-expressing cells confirmed an increased nuclear association of ATR-pS435 and XPA following cisplatin treatment (Fig. 5A,B). In contrast, *MC1R* ^*WT*^-expressing cells pre-treated with the MC1R antagonists ASIP or HBD3 failed to exhibit MSH-induced increases in ATR-pS435-XPA association (Fig. 5A,B). Incubation of MSH enhanced the interaction between XPA and cisplatin-adducts compared to vehicle (Fig. S9). In contrast, incubation with either ASIP or HBD3 antagonized MSH’s enhancement of the co-localization of XPA and cisplatin adducts. Taken together, these data indicate that cAMP signaling enhances interactions of ATR-pS435 and XPA to cisplatin-damaged chromatin.

RETRACTED

**Figure 5:** MC1R-cAMP signaling promotes XPA-ATR-pS435 interactions following cisplatin-induced DNA damage. (**A**) XPA-ATR-pS435 interactions were determined by proximity ligation using anti-XPA and anti-ATR-pS435 antibodies. Wild-type MC1R expressing HEK293 cells were pre-treated with MSH (100 nM), MSH (100 nM) + ASIP (100 nM) or MSH (100 nM) + HBD3 (100 nM) 30 minutes before cisplatin treatment (100 µM) for 1 hr. Green detection events signify juxtaposition between XPA and ATR-pS435 in maximum intensity projection images 30 min after cisplatin exposure. Nuclei were stained with DAPI (blue). Bar represents 50 µm. (**B**) Quantification of the XPA-ATR-pS435 colocalization shown in panel B. At least 100 cells were counted from representative fields from two separate experiments and extent of interaction is expressed as fold-change compared to undamaged cells obtained from maximum intensity images from focal plane z-stacks. Values not sharing a common letter were significantly different as determined by one-way ANOVA; p ≤ 0.05. Data are expressed as mean ± SEM.

### MC1R/cAMP suppresses cisplatin-induced mutagenesis

Since we had already observed that cAMP signaling induced ATR-pS435 accumulation, promoted its co-localization with XPA on cisplatin-damaged chromatin and accelerated clearance of cisplatin intrastrand DNA adducts, we reasoned that MC1R/cAMP signaling protects melanocytes against cisplatin-induced mutagenesis. To determine this, we quantified the impact of MC1R agonists and antagonists on cisplatin-induced mutational rate using the *HPRT* mutagenesis assay^43^. Pretreating PHMs and HEK293 cells expressing wild-type MC1R with MSH or forskolin resulted in marked reductions in cisplatin-induced mutagenesis (Fig. 6A,B). Co-treatment of either cell type with HBD3 or ASIP blocked MSH- but not forskolin-mediated protection against cisplatin-mediated mutagenesis (Fig. 6A,B). In contrast, in an MC1R-dysfunctional setting (HEK293 cells expressing MC1R^*R151C*^), MSH failed to protect against cisplatin mutagenesis (Fig. S10). Taken together, our studies confirm that MC1R/cAMP signaling enhances the repair of cisplatin-mediated DNA damage, reduces cisplatin-induced mutagenesis and support the concept that cAMP induction may be a viable anti-mutagenic strategy against cisplatin-mediated DNA damage.

**Figure 6:** MC1R-cAMP signaling protects against cisplatin-induced mutagenesis. (**A**) PHM or (**B**) *MC1R* ^*WT*^-expressing HEK293 cells pre-treated with either forskolin (10 µM), MSH (100 nM), MSH (100 nM) + ASIP (100 nM) or MSH (100 nM) + HBD3 (100 nM) 30 minutes before cisplatin treatment (100 µM) for 1 hr. Colony-forming efficiency was determined at 21 days post-6-TG treatment. Note: no colonies were observed in the absence of cisplatin-induced damage. Values not sharing a common letter are significantly different as determined by Poisson regression analysis (*p* ≤ 0.05). Data shown are representative of two independent experiments with each experiment containing six biological replicates.

RETRACTED

## Discussion

The melanocortin 1 receptor (MC1R) is a G_s_ protein coupled receptor expressed on melanocytes that regulates many aspects of melanocyte physiology^7,44^. Loss-of-function MC1R polymorphisms are common and clearly increase lifetime melanoma risk^6^. In addition to influencing the amount and type of melanin made by melanocytes^45^, MC1R signaling, mediated by the second messenger cAMP, controls how efficiently melanocytes respond to cell damage^8,46^. MC1R signaling enhances the efficiency of nucleotide excision repair (NER), the maintenance pathway charged with the removal of mutagenic UV photoproducts and other bulky adducts from genomic DNA^20,47^. We previously reported that a key molecular event linking MC1R signaling to NER is cAMP-induced activation of PKA, which then phosphorylates ATR on the S435 residue and leads to recruitment of the NER factor XPA and co-localization of the ATR-pS435-XPA complex to sites of UV photodamage to enhance NER^19^. Subsequently, we found that AKAP12 functions as a critical molecular scaffold required for PKA-mediated generation of ATR-pS435 and that the mechanism by which cAMP enhances NER is through accelerated 5′ strand incision^41^. Our prior studies addressed the mechanisms by which MC1R signaling influences repair of UV photodamage, however the impact this cAMP-mediated system may have against other mutagenic DNA lesions remained unexplored.

Hypothesizing that MC1R/cAMP-enhanced NER may extend to other forms of DNA injury besides UV damage, we evaluated the effect of cAMP signaling on melanocyte responses to cisplatin, a platinum-containing chemotherapeutic that forms helix-distorting lesions via both intra- and inter-strand cross links^48^. More than 90% of DNA adducts formed by cisplatin are intrastrand cross-links including 1,2-d(GpG) cross-links, which are repaired by NER^49^. By using an intrastrand lesion-specific cisplatin-DNA antibody that recognizes 1,2-d(GpG) cross-links, we were able to precisely measure the repair kinetics of cisplatin-damaged DNA. We found that induction of cAMP signaling, either physiologically induced through MSH-MC1R signaling or pharmacologically by forskolin, robustly accelerated the clearance of cisplatin-induced DNA adducts in PHMs and in MC1R-expressing HEK293 cells. MSH-enhanced clearance of cisplatin DNA damage was inhibited by MC1R antagonists HBD3 and ASIP, supporting the hypothesis that repair of cisplatin-damaged DNA is regulated through MC1R-ligand interactions. Forskolin, an agent that potently induces cAMP by directly activating adenylyl cyclase, overcame signaling defects caused by defective MC1R or the presence of MC1R antagonists, suggesting that pharmacologic induction of cAMP signaling may be useful to enhance melanocyte genomic stability against cisplatin damage. Comparing our current findings with prior studies^19,41^, we noted greater cAMP-mediated enhancement of cisplatin damage than for UV photolesions. This may indicate differential cAMP repair profiles for distinct DNA lesions, perhaps explained by variable conformational alterations in DNA, biological activities and/or extent of lesions generated by damaging agents.

RETRACTED

To elucidate the mechanistic effect of MC1R ligands on the repair of cisplatin DNA adducts, we adapted the oligonucleotide retrieval immunoprecipitation (ORiP) assay^39,41^ but instead of incorporating UV damage as “bait”, we generated a cisplatin-exposed oligonucleotide construct to study kinetics of association between repair proteins and cisplatin-damaged DNA. Using this assay, we found increased association of several NER-enhancing proteins in the cAMP repair axis with cisplatin-damaged DNA including ATR, ATR-pS435, AKAP12 and XPA. One caveat to interpretation of ORiP data, however, is that binding between proteins of interest and DNA may be due to multiple reasons besides increased affinity including differential protein levels, uncharacterized protein-protein interactions or other post-translational modifications. Nonetheless, we documented that cisplatin damage repair and interactions of ATR, ATR-pS435, AKAP12 and XPA with cisplatin-damaged DNA were each regulated by MC1R signaling and appropriate receptor-ligand interactions. While our previous studies focused on XPA’s association with UV photodamage^50^, data presented here link cAMP signaling with efficiency of XPA recruitment to cisplatin-damaged DNA. Given the essential role of XPA in DNA repair and genome maintenance^51,52^, our findings suggest that MC1R/cAMP-mediated XPA interactions may be an important cellular strategy to reduce risk of mutagenesis to a range of NER substrates.

Our previous work established that the critical molecular event needed for improvement of NER by cAMP signaling is PKA-mediated ATR phosphorylation on the S435 residue^19^, however this does not occur to any appreciable extent in undamaged cells. Therefore, in addition to cAMP signaling, there must be cellular damage signals to appropriately activate ATR. Using a phospho-specific antibody that recognizes ATR-pS435, we performed enzyme kinetic studies to study ATR-pS435 kinetics after cisplatin exposure and found that cAMP induction yielded higher V_max_ and lower K_m_ values for ATR-pS435 accumulation. Physiologically, cAMP may enhance the capability of PKA to recognize ATR-S435 and/or impact how strongly PKA interacts with the S435 residue. In any case, our current studies establish that cisplatin is a robust signal for ATR to become a substrate for PKA to enable cAMP-enhanced repair.

RETRACTED

Our data suggest PKA-cAMP-signaling favors enhancement of XPA to NER-relevant damage^19,41^. Interestingly, we did not observe any effect of cAMP on association of XPC or CSB with UV-damaged chromatin, suggesting that cAMP-mediated NER enhancement lies downstream of damage recognition. As XPA is a core factor in both TCR- and GGR, an XPA-driven mechanism could potentially enable a cAMP boost to both TCR and GGR^20^. In addition, acute and chronic PKA-cAMP signaling might involve differential UV responses. These mechanisms may have evolved to ensure long term genomic stability and prevent melanoma formation. Collectively, short-term cAMP signaling (minutes to hours) may involve post-translational modifications of certain repair proteins, while prolonged cAMP-signaling (several days) could also regulate transcriptional and translational responses to damage^14,18,19,44^.

We also explored the impact of cAMP signaling on the repair of DNA damage induced by other platinum compounds. Using XL-PCR, we observed distinct repair profiles between cisplatin, oxaliplatin, carboplatin and phenanthriplatin, possibility related to the respective DNA helical-distortion each agent generates^53–55^. Nonetheless, cAMP signaling enhanced repair of both traditional bi-functional platinum compounds (cisplatin, oxaliplatin, carboplatin) and nonclassical mono-functional agents (phenanthriplatin), supporting the concept of pharmacologic cAMP activation as a strategy for enhanced melanocyte genomic stability against a variety of platinum compounds.

Finally, we found that cAMP markedly reduced cisplatin-mediated mutagenesis in melanocytes, suggesting that melanocyte-directed cAMP induction may be a useful strategy to reduce risk of secondary melanomas in cisplatin-treated cancer patients, particularly among “high-risk” individuals with inherited defects in MC1R known to predispose to melanomas^6,56^. Recent reports confirm that inheritance of even one abnormal MC1R allele is associated with a higher mutagenic burden in melanoma^57^, strongly suggesting a link between MC1R function and DNA repair. In addition, loss-of-function mutations in ATR occur in a subset of melanomas with a higher somatic mutational load^35^. Together, our findings support the hypothesis that MC1R/cAMP signals coupled with ATR-dependent events regulate melanocytic NER, reduce cisplatin-induced mutagenesis and raise the possibility that pharmacologic cAMP activation may be a useful strategy for enhanced melanocyte genomic stability to reduce secondary melanoma risk in patients treated with platinum-containing chemotherapeutics.

RETRACTED

## Methods

### Cell lines, plasmids, recombinant proteins, siRNA and cisplatin-induced damage

Transformed cell lines HEK293 (ATCC) and melanocytes (Coriell) were cultured in RPMI-10% FBS media. HEK293 cells were transfected with either MC1R-WT, MC1R-R151C, AKAP12-WT or AKAP12^ΔPKA^ as described^19,41^. pcDNA3.1 vectors containing either wild-type ATR^58^ or mutated ATR (S435A)^19^ were used as previously described. All transfections and siRNA knockdowns were confirmed by Western blotting. Recombinant MSH (Sigma), ASIP (BD Biosciences) and HBD3 (BD Biosciences) were used as indicated. siRNA targeted to ATR and AKAP12 (Dharmacon) was performed using manufacturer’s instructions. All platinum agents were used at a concentration of 100 µM for cell culture studies.

### Antibodies

Antibodies used were ATR-pS435 and ATR-WT^19^, AKAP12 (Thermo Fisher Scientific, Cat #PA5-21759), Pt-GpG (Abcam, Cat #103261), XPA (Cell Signaling, Cat #14607 S), XPC (Cell Signaling, Cat #14768), CSB (Bethyl, Cat #A301), H2A (Cell Signaling, Cat #12349), tubulin (Santa Cruz, Cat #sc-9104).

### DNA repair kinetics and mutagenesis

Cells were exposed to platinum agents (cisplatin, oxaliplatin, carboplatin and phenanthriplatin; 100 µM) for 1 hr, followed by two PBS washes and re-addition of RPMI media for indicated times. Immuno-slot blots were performed with an intrastrand lesion-specific cisplatin-DNA antibody (anti-Pt-GpG) using standard slot-blot protocols. Presence of platinum-induced DNA polymerase-blocking lesions was assessed using XL-PCR, repair of a 5 kb fragment of the *HPRT* gene was assessed by PCR 5′-CCCAACTCACCACAACCTCT-3′ and 5′-AGGGAACCCTTCTGTGTGTG-3′, essentially as described^38^. Efficiency of PCR amplification between damage and control samples was used to calculate repair at each time point as described. The frequencies of cisplatin-induced *HPRT* mutations were measured as previously described^41^.

### Sub-cellular fractionation, immunoprecipitation and immunoblotting

Sub-cellular fractionation was performed with ∼2 × 10^6^ cells, washed with PBS and resuspended in 200 μL of solution A (10 mM HEPES at pH 7.9, 10 mM KCl, 1.5 mM MgCl_2_, 0.34 M sucrose, 10% glycerol, 1 mM DTT, and protease inhibitors (Halt Protease and Phosphatase inhibitors; Thermo Scientific). Cells were lysed with Triton X-100 (0.05%). Cytoplasmic proteins were separated from nuclei by centrifugation at 1000 *g* for 5 min. Isolated nuclei were washed with solution A and lysed in 200 μL of solution B (3 mM EDTA, 0.2 mM EGTA, 1 mM DTT). The soluble nuclear proteins were separated from chromatin by centrifugation at 2000*g* for 5 min. To release the proteins associated with DNA for ORiP assays, the pellet was treated with DNase I (50 U) for 30 min at 37 °C in 60 mM Tris-HCl (pH 7.5), 2.5 mM MgCl_2_ and, 11 mM CaCl_2_). The reaction was stopped by the addition of 1 mM EGTA and the reaction centrifuged at 2000 g for 5 min at 4 °C to obtain the supernatant. To obtain chromatin containing proteins for Western blotting, the chromatin pellet was washed once with solution B and centrifuged at 10,000 *g* for 1 min. Isolated chromatin was resuspended in 20 mM Tris-HCl, pH 7.9, 100 mM NaCl, 20% glycerol, 0.1 Nonidet P-40 and sheared by sonication. Chromatin-bound proteins were obtained after centrifugation at 10,000 g for 10 min. Samples were resuspended in 100 μL of SDS sample buffer and heated at 95 °C for 10 min before Western analysis. For Western Blot acquisition analysis, a Storm 860 was used and Western blots scanned using channel 2 with blue excitation at 450 nm and emission at 520 nm, sensitivity was set to normal and PMT voltage set to 400 V.

RETRACTED

### ATR-pS435 detection and enzyme kinetics

ATR-S435 kinase assays were performed using a biotinylated ATR peptide substrate, CPKRRRLSSSLNPS (Genscript). The peptide was previously validated as specific to S435 phosphorylation in the context of a 14-mer ATR peptide^39^. The kinetic parameters of the phosphorylation reaction were calculated by nonlinear regression analysis with GraphPad Prism.

### Oligonucleotide retrieval-immunoprecipitation (ORiP)

Synthetic oligonucleotides (Molecular Beacons) were assembled to form 5′-biotinylated duplex DNA fragments that acts as substrates for NER proteins. A 30-nt oligonucleotide, 5′-CTCGTCAGCATCTTCATCATACAGTCAGTG-3′, was allowed to react at a concentration of 1 mM cisplatin for 16 h at 37 °C in a buffer containing 3 mM NaCl, 0.5 mM of Na_2_HPO_4_ and NaH_2_PO_4_. After ethanol precipitation, the oligo was annealed and ligated with two oligonucleotides, as previously described^39^. After indicated treatments, extracts (50 µg) were incubated with the biotinylated oligonucleotide in streptavidin-coated 96 well plates (Thermo-Scientific) (0.01 nM per well) for indicated times at 30 °C. Wells were washed with 40 mM Tris-HCl (pH 7.5) containing 0.01% BSA (wash buffer) followed by fixation in 4% paraformaldehyde. Indicated antibodies (either anti-XPA, anti-ATR, anti-AKAP12) (2 µg) was added for 1 h and detection accomplished using 1-Step Ultra TMB ELISA Substrate (Pierce) with absorbance measured at 400 nm.

RETRACTED

### Immunofluorescence, ***in situ*** detergent extraction and proximity ligation assay

Following cisplatin damage, cells were either processed immediately, or medium was replaced and DNA repair allowed for indicated periods. Cell extraction was carried out *in situ* by washes of 0.1% Nonidet P-40 for 10 minutes on ice to remove all soluble proteins. Following fixation in 4% paraformaldehyde and cell permeabilization with 0.3% Triton X-100, cells were blocked overnight in 10% donkey serum at 4 °C. After incubation with indicated primary and secondary antibodies, cells were mounted with Prolong Gold antifade. Proximity ligation assay (DuoLink, Sigma) was performed using the manufacturer’s instructions. All fluorescence images were obtained using a Leica DMI 6000 confocal microscope using ×100 objective (1.4 numerical aperture) with LAS AF 2.7.2.9586 software (Leica Application Suite Advanced Fluorescence). Maximum intensity images from focal plane z-stacks (spaced 0.2 µm apart) were acquired and deconvoluted. Quantification of fluorescent signal were performed using Image J software.

### Statistical Analysis

Student’s t tests, and one-way ANOVA were performed with GraphPad Prism 5.0. Poisson regression analysis was performed using SAS software. Data were considered statistically significant if p values were less than 0.05.

## Electronic supplementary material

Supplementary Data

## References

[1] Shahrokni A, Wu AJ, Carter J, Lichtman SM (2016). Long-term Toxicity of Cancer Treatment in Older Patients. Clin Geriatr Med.

[2] Pappo, A. S. Melanoma in children and adolescents. *Eur J Cancer***39**, 2651–2661, doi:S0959804903006944 (2003).10.1016/j.ejca.2003.06.00114642927

[3] Sharma D, Lee T, Friedman AJ, Redbord KP (2017). Need For Improved Skin Cancer Surveillance in Pediatric Cancer Survivors. Am J Clin Dermatol.

[4] Bucci, B. *et al*. Myc down-regulation sensitizes melanoma cells to radiotherapy by inhibiting MLH1 and MSH2 mismatch repair proteins. *Clin Cancer Res***11**, 2756–2767, doi:11/7/2756 (2005).10.1158/1078-0432.CCR-04-158215814658

[5] Braam KI (2012). Malignant melanoma as second malignant neoplasm in long-term childhood cancer survivors: a systematic review. Pediatr Blood Cancer.

RETRACTED

[6] Valverde P, Healy E, Jackson I, Rees JL, Thody AJ (1995). Variants of the melanocyte-stimulating hormone receptor gene are associated with red hair and fair skin in humans. Nat Genet.

[7] Wolf Horrell EM, Boulanger MC, D’Orazio JA (2016). Melanocortin 1 Receptor: Structure, Function, and Regulation. Frontiers in genetics.

[8] Kadekaro, A. L. *et al*. Melanocortin 1 receptor genotype: an important determinant of the damage response of melanocytes to ultraviolet radiation. *Faseb J*, doi:fj.10-158485 (2010).10.1096/fj.10-158485PMC322942120519635

[9] Suzuki I, Cone RD, Im S, Nordlund J, Abdel-Malek ZA (1996). Binding of melanotropic hormones to the melanocortin receptor MC1R on human melanocytes stimulates proliferation and melanogenesis. Endocrinology.

[10] Suzuki, I. *et al*. Agouti signaling protein inhibits melanogenesis and the response of human melanocytes to alpha-melanotropin. *J Invest Dermatol***108**, 838–842, doi:S0022202X97862847 (1997).10.1111/1523-1747.ep122925729182807

[11] Candille SI (2007). A -defensin mutation causes black coat color in domestic dogs. Science.

[12] Nix MA (2013). Molecular and functional analysis of human beta-defensin 3 action at melanocortin receptors. Chem Biol.

[13] Garcia-Borron JC, Abdel-Malek Z, Jimenez-Cervantes C (2014). MC1R, the cAMP pathway, and the response to solar UV: extending the horizon beyond pigmentation. Pigment Cell Melanoma Res.

[14] Wong, S. S., Ainger, S. A., Leonard, J. H. & Sturm, R. A. MC1R variant allele effects on UVR-induced phosphorylation of p38, p53, and DDB2 repair protein responses in melanocytic cells in culture. *J Invest Dermatol***132**, 1452–1461, doi:jid2011473 (2012).10.1038/jid.2011.47322336944

[15] Bowden NA (2013). Regulators of global genome repair do not respond to DNA damaging therapy but correlate with survival in melanoma. PLoS One.

[16] Smith AG (2008). Melanocortin-1 receptor signaling markedly induces the expression of the NR4A nuclear receptor subgroup in melanocytic cells. J Biol Chem.

[17] Kadekaro, A. L. *et al*. Alpha-melanocyte-stimulating hormone suppresses oxidative stress through a p53-mediated signaling pathway in human melanocytes. *Mol Cancer Res***10**, 778–786, doi:1541-7786.MCR-11-0436 (2012).10.1158/1541-7786.MCR-11-043622622028

[18] Swope V (2014). Significance of the melanocortin 1 receptor in the DNA damage response of human melanocytes to ultraviolet radiation. Pigment Cell Melanoma Res.

[19] Jarrett SG (2014). PKA-mediated phosphorylation of ATR promotes recruitment of XPA to UV-induced DNA damage. Mol Cell.

[20] Scharer OD (2013). Nucleotide excision repair in eukaryotes. Cold Spring Harb Perspect Biol.

RETRACTED

[21] Kraemer KH (2007). Xeroderma pigmentosum, trichothiodystrophy and Cockayne syndrome: a complex genotype-phenotype relationship. Neuroscience.

[22] Kraemer KH (1990). Defective DNA repair in humans: clinical and molecular studies of xeroderma pigmentosum. Basic Life Sci.

[23] Kraemer KH, Tamura D, Khan SG, Digiovanna JJ (2013). Burning issues in the diagnosis of xeroderma pigmentosum. Br J Dermatol.

[24] Lehmann AR (2003). DNA repair-deficient diseases, xeroderma pigmentosum, Cockayne syndrome and trichothiodystrophy. Biochimie.

[25] Lehmann, A. R., McGibbon, D. & Stefanini, M. Xeroderma pigmentosum. *Orphanet J Rare Dis***6**, 70, doi:1750-1172-6-70 (2011).10.1186/1750-1172-6-70PMC322164222044607

[26] Krasikova YS, Rechkunova NI, Maltseva EA, Petruseva IO, Lavrik OI (2010). Localization of xeroderma pigmentosum group A protein and replication protein A on damaged DNA in nucleotide excision repair. Nucleic Acids Res.

[27] Matsuda T (1995). DNA repair protein XPA binds replication protein A (RPA). J Biol Chem.

[28] Matsuoka S (2007). ATM and ATR substrate analysis reveals extensive protein networks responsive to DNA damage. Science.

[29] Lindsey-Boltz, L. A., Sercin, O., Choi, J. H. & Sancar, A. Reconstitution of human claspin-mediated phosphorylation of Chk1 by the ATR (ataxia telangiectasia-mutated and rad3-related) checkpoint kinase. *J Biol Chem***284**, 33107–33114, doi:M109.064485 (2009).10.1074/jbc.M109.064485PMC278515219828454

[30] Munoz MJ (2017). Major Roles for Pyrimidine Dimers, Nucleotide Excision Repair, and ATR in the Alternative Splicing Response to UV Irradiation. Cell Rep.

[31] Belanger F, Rajotte V, Drobetsky EA (2014). A majority of human melanoma cell lines exhibits an S phase-specific defect in excision of UV-induced DNA photoproducts. PLoS One.

[32] Li Z, Musich PR, Cartwright BM, Wang H, Zou Y (2013). UV-induced nuclear import of XPA is mediated by importin-alpha4 in an ATR-dependent manner. PLoS One.

[33] Wu, X., Shell, S. M., Liu, Y. & Zou, Y. ATR-dependent checkpoint modulates XPA nuclear import in response to UV irradiation. *Oncogene***26**, 757–764, doi:1209828 (2007).10.1038/sj.onc.1209828PMC310610416862173

[34] Lee TH, Park JM, Leem SH, Kang TH (2014). Coordinated regulation of XPA stability by ATR and HERC2 during nucleotide excision repair. Oncogene.

[35] Chen CF (2017). ATR Mutations Promote the Growth of Melanoma Tumors by Modulating the Immune Microenvironment. Cell Rep.

[36] Kadekaro AL, Kanto H, Kavanagh R, Abdel-Malek Z (2003). Significance of the melanocortin 1 receptor in regulating human melanocyte pigmentation, proliferation, and survival. Ann N Y Acad Sci.

[37] Kadekaro AL (2005). alpha-Melanocortin and endothelin-1 activate antiapoptotic pathways and reduce DNA damage in human melanocytes. Cancer Res.

RETRACTED

[38] Ayala-Torres S, Chen Y, Svoboda T, Rosenblatt J, Van Houten B (2000). Analysis of gene-specific DNA damage and repair using quantitative polymerase chain reaction. Methods.

[39] Jarrett SG, Wolf Horrell EM, Boulanger MC, D’Orazio JA (2015). Defining the Contribution of MC1R Physiological Ligands to ATR Phosphorylation at Ser435, a Predictor of DNA Repair in Melanocytes. J Invest Dermatol.

[40] Johnstone, T. C., Suntharalingam, K. & Lippard, S. J. Third row transition metals for the treatment of cancer. *Philos Trans A Math Phys Eng Sci***373**, doi:10.1098/rsta.2014.0185 (2015).10.1098/rsta.2014.0185PMC434297325666060

[41] Jarrett SG, Wolf Horrell EM, D’Orazio JA (2016). AKAP12 mediates PKA-induced phosphorylation of ATR to enhance nucleotide excision repair. Nucleic Acids Res.

[42] Kang TH, Reardon JT, Sancar A (2011). Regulation of nucleotide excision repair activity by transcriptional and post-transcriptional control of the XPA protein. Nucleic Acids Res.

[43] Glaab WE, Tindall KR (1997). Mutation rate at the hprt locus in human cancer cell lines with specific mismatch repair-gene defects. Carcinogenesis.

[44] Swope VB, Abdel-Malek ZA (2016). Significance of the Melanocortin 1 and Endothelin B Receptors in Melanocyte Homeostasis and Prevention of Sun-Induced Genotoxicity. Frontiers in genetics.

[45] Barsh G, Gunn T, He L, Schlossman S, Duke-Cohan J (2000). Biochemical and genetic studies of pigment-type switching. Pigment Cell Res.

[46] Abdel-Malek, Z. A., Knittel, J., Kadekaro, A. L., Swope, V. B. & Starner, R. The melanocortin 1 receptor and the UV response of human melanocytes–a shift in paradigm. *Photochem Photobiol***84**, 501–508, doi:PHP294 (2008).10.1111/j.1751-1097.2008.00294.x18282187

[47] Marteijn JA, Lans H, Vermeulen W, Hoeijmakers JH (2014). Understanding nucleotide excision repair and its roles in cancer and ageing. Nat Rev Mol Cell Biol.

[48] Eastman A (1985). Interstrand cross-links and sequence specificity in the reaction of cis-dichloro(ethylenediamine)platinum(II) with DNA. Biochemistry.

[49] Jamieson ER, Lippard SJ (1999). Structure, Recognition, and Processing of Cisplatin-DNA Adducts. Chem Rev.

[50] Lindsey-Boltz LA (2014). Coupling of human DNA excision repair and the DNA damage checkpoint in a defined *in vitro* system. J Biol Chem.

[51] Cimprich, K. A. & Cortez, D. ATR: an essential regulator of genome integrity. *Nat Rev Mol Cell Biol***9**, 616–627, doi:nrm2450 (2008).10.1038/nrm2450PMC266338418594563

[52] Sirbu, B. M. & Cortez, D. DNA damage response: three levels of DNA repair regulation. *Cold Spring Harb Perspect Biol***5**, doi:10.1101/cshperspect.a012724 (2013).10.1101/cshperspect.a012724PMC372127823813586

RETRACTED

[53] Park GY, Wilson JJ, Song Y, Lippard SJ (2012). Phenanthriplatin, a monofunctional DNA-binding platinum anticancer drug candidate with unusual potency and cellular activity profile. Proc Natl Acad Sci USA.

[54] Spingler B, Whittington DA, Lippard SJ (2001). 2.4 A crystal structure of an oxaliplatin 1,2-d(GpG) intrastrand cross-link in a DNA dodecamer duplex. Inorg Chem.

[55] Teuben JM, Bauer C, Wang AH, Reedijk J (1999). Solution structure of a DNA duplex containing a cis-diammineplatinum(II) 1,3-d(GTG) intrastrand cross-link, a major adduct in cells treated with the anticancer drug carboplatin. Biochemistry.

[56] Valverde P (1996). The Asp84Glu variant of the melanocortin 1 receptor (MC1R) is associated with melanoma. Hum Mol Genet.

[57] Robles-Espinoza CD (2016). Germline MC1R status influences somatic mutation burden in melanoma. Nat Commun.

[58] Jiang, G. & Sancar, A. Recruitment of DNA damage checkpoint proteins to damage in transcribed and nontranscribed sequences. *Mol Cell Biol***26**, 39–49, doi:26/1/39 (2006).10.1128/MCB.26.1.39-49.2006PMC131763716354678

